# Preliminary Evaluation of the Value of a Small‐Molecule Probe Targeting DNMT1 in Detecting the Methylation of PAX1 in Cervical Cancer

This article has been retracted.

**DOI:** 10.1111/srt.70074

**Published:** 2024-09-27

**Authors:** Baohua Yang, Qunxian Cheng, Xiaoqian Hong, Xiuxiang Zhu, Ziyin Xia, Wei Chen, Ling Xu

**Affiliations:** ^1^ Department of Obstetrics and Gynecology Minhang Hospital Fudan University Shanghai China; ^2^ Department of Medicinal Chemistry School of Pharmacy Fudan University Shanghai China

**Keywords:** assessment, cervical cancer, methylation marker, screening value, small molecule probe

## Abstract

**Background:**

To investigate the screening value of a small‐molecule probe to assess the methylation of PAX1 in cervical cancer.

**Materials and Methods:**

The diagnostic threshold of the grayscale values for cervical lesions was assessed by plotting the Receiver Operating Characteristic (ROC) curve of subjects. Grayscale values were significantly different among the four groups (*p* < 0.05). Compared with the LSIL and cervicitis groups, a considerably higher grayscale value was found in the CA and high‐grade squamous intraepithelial lesion (HSIL) groups (both *p* < 0.05).

**Results:**

The differential ROC curves of the grayscale values showed that the diagnostic Area Under Curve of the probe for cervicitis and low‐grade squamous intraepithelial lesion (LSIL) was 0.8724 (95% CI = 0.7762–0.9685, *p* < 0.0001), for cervicitis and CA was 1.0000 (*p* < 0.0001), for the LSIL and HSIL was 0.5484 (95% CI = 0.3826–0.7142, *p* = 0.5755), and for the LSIL and CA was 0.7724 (95% CI = 0.6016–0.9432, *p* = 0.0138).

**Conclusion:**

The small molecular probe has certain application value in differentiating the type of cervical lesions and has better efficacy in distinguishing cervical inflammatory and precancerous lesions from carcinogenesis, but less efficacy in determining the type of precancerous lesions.

## 1 Introduction

Cervical cancer incidence is second only to breast cancer, ranking second in the incidence of female malignant tumors [1]. With the change in lifestyle and daily habits of residents in recent years, statistics shows that there are about 500,000 new cases of cervical cancer and 231,000 deaths each year worldwide. The annual incidence of cervical cancer in China is as high as 131,500, and its incidence and mortality rank first among female malignant tumors in China [2, 3]. Viral infection, multiple deliveries, smoking, and other factors may induce cervical cancer. Because the clinical symptoms of early cervical cancer are not obvious, most patients have developed cervical cancer to the middle and late stages at the time of detection, and the healing of cervical cancer at this stage mainly includes surgical healing, chemotherapy, and radiotherapy [4, 5]. Early diagnosis and intervention of cervical cancer are important means to enhance the prognosis of patients, and it is also of great significance to develop individualized healing plans [6].

Molecular biology technology is being increasingly used in cancer screening. Some scholars have found that DNA methylation is prevalent in cervical exfoliated cells, cervical biopsy tissues, and plasma samples [6, 7]. At present, the continuous development and maturity of protein labeling technology have led to the discovery of the application value of protein fluorescence analysis in cancer screening, and the small‐molecule fluorescence probe technology can achieve visualization and tracer monitoring through the labeling of proteins [8, 9]. In this study, we will analyze the screening value of a small‐molecule probe in assessing the methylation of a cervical cancer marker PAX1, providing a reference for improving the prognosis of patients with cervical cancer.

## 2 Materials and Methods

### 2.1 General Data

Eighty‐one cervical tissues from patients, who visited our cervical specialist clinic from August 2020 to January 2022, were enrolled and quantitatively tested for methylation of the tumor suppressor gene PAX1 after liquid nitrogen preservation, and the pathological test results were used as the gold standard to distinguish them into the cervicitis group (*n* = 23), low‐grade squamous intraepithelial lesion (LSIL, *n* = 31), high‐grade squamous intraepithelial lesion (HSIL, *n* = 18), and cervical cancer group (CA, *n* = 9).

Inclusion criteria were (1) clinical medical records were complete and (2) the investigation was approved by the Ethics Association of the hospital.

Exclusion criteria were (1) patients with other malignant tumors, (2) patients with mental illness, (3) patients who were ongoing other clinical research, and (4) drug‐ or alcohol‐dependent individuals.

### 2.2 Quantitative Detection of DNMT1 in Cervical Tissue by a Small‐Molecule Fluorescent Probe

PAX1 methylation is mainly mediated by DNA methyltransferase 1 (DNMT1), which plays an important role as a PAX1 methylation promoter in cervical cancer cells. Our group collaborating with the Pharmaceutical Chemistry Laboratory of Fudan University has designed and synthesized a small‐molecule fluorescent probe RG108‐FITC (Patent number: CN201910750081.X) deriving from the combination of ligand or inhibitor of DNMT1 and a specific fluorescent group. The probe is capable of determining the level of DNMT1 in cells by specifically binding to DNMT1, thereby indirectly determining the methylation level of PAX1. For the DNMT1 fluorescence quantitative assay, after centrifuging the cell suspension, the cells were diluted with medium, counted, and transferred to a new centrifuge tube. An appropriate amount of culture solution containing the probe was then added until the total liquid volume reached 1 mL. Subsequently, the cells were collected after incubation at 37°C for 4 h, followed by nuclear staining with DAPI (0.1 ug/mL) for 10 min. Images of DAPI and fluorescent probe were obtained by confocal fluorescence microscopy (Nikon) at 349 and 488 nm, respectively. The fluorescence intensity was calculated by ImageJ.

### 2.3 Outcome Measurements

The primary outcome was the efficacy of the probe in distinguishing various cervical lesions. Applying the pathological results as the gold standard, the grayscale values of different cervical lesions were detected. After the comparison of the grayscale values, the Receiver Operating Characteristic (ROC) curve was plotted and therefore the diagnostic efficacy of the probe to distinguish different cervical lesions was evaluated based on the curse.

### 2.4 Statistical Methods

The results were expressed as median and quartiles, and the diagnostic value of the grayscale values for different cervical lesions was plotted by ROC curve. Variances were considered remarkable at *p* < 0.05. GraphPad Prism 8.3 was used for plotting.

## 3 Results

### 3.1 Comparison of the Grayscale Values of Different Cervical Lesion Tissues

A remarkable significance was indicated by the comparison of the grayscale values for all groups (*p* < 0.05). In comparing the two groups, the grayscale value in the CA group was prominently higher than the LSIL and cervicitis groups (*p* < 0.05), and the grayscale value in the HSIL group was notably superior to the LSIL and cervicitis groups (*p* < 0.05). Table 1 shows a comparison of the grayscale values of the small‐molecule probe in different cervical lesions, Figure 1 shows a comparison of the greyscale values of the small‐molecule probe in different cervical lesions.

**TABLE 1:** Comparison of the grayscale values of the small‐molecule probe in different cervical lesions ($\bar{x}\pm s$).

Groups	Cases	Grayscale values
Cervicitis	23	24.88 ± 13.39
LSIL	31	61.30 ± 23.18
HSIL	18	71.62 ± 12.60^ab^
CA	9	78.91 ± 8.22^ab^
*t*	—	34.477
*p*	—	<0.001

*Note*: ^a^ represents *p* < 0.05, compared to the cervicitis group, and ^b^ represents *p* < 0.05, compared to the LSIL group.

**FIGURE 1:** Comparison of the grayscale values of the small‐molecule probe in different cervical lesions. A remarkably higher grayscale value was indicated in the CA group compared with the cervicitis and LSIL groups. Compared to the cervicitis and LSIL groups, the HSIL group exhibited a noticeably greater grayscale value.

### 3.2 Analysis of the Grayscale Values of the Small‐Molecule Probe in Differentiating Cervical Lesions

ROC curves were plotted for the differentiation of different cervical lesions by the grayscale values of the probe, and the results suggested that the diagnostic Area Under Curve (AUC) of the grayscale values of the probe was 0.8724 (95% CI = 0.7762−0.9685, *p* < 0.0001) for the cervicitis and LSIL groups, 1.0000 (*p* < 0.0001) for cervicitis and HSIL, and 1.0000 (*p* < 0.0001) for cervicitis and CA, as shown in Table 2 and Figure 2. The diagnostic AUC of the probe was 0.5484 (95% CI = 0.3826−0.7142, *p =* 0.5755) for LSIL versus HSIL, 0.7724 (95% CI = 0.6016−0.9432, *p =* 0.0138) for LSIL versus CA, as shown in Figure 3, and 0.7037 (95% CI = 0.4639−0.9435, *p =* 0.0896) for HSIL versus CA, as shown in Figure 4.

**TABLE 2:** Analysis of the grayscale values of the small‐molecule probe in differentiating cervical lesions.

Types of diagnosis	AUC	SE	95% CI	*p*
Cervicitis and LSIL	0.8724	0.049	0.7762–0.9685	*p* < 0.001
Cervicitis with HSIL	1.000	0.000	1.000–1.000	*p *< 0.001
Cervicitis with CA	1.000	0.000	1.000–1.000	*p* < 0.001
LSIL with HSIL	0.5484	0.085	0.3826–0.7142	0.5755
LSIL with CA	0.7724	0.087	0.6016–0.9432	0.0138
HSIL and CA	0.7037	0.122	0.4639–0.9435	0.0896

Abbreviations: AUC, Area Under Curve.

**FIGURE 2:** The diagnostic ROC curves of the grayscale values of the small‐molecule probe for cervicitis versus LSIL, HSIL, and CA. The diagnostic AUC of the small‐molecule probe grayscale values for cervicitis versus LSIL was 0.8724 (95% CI = 0.7762–0.9685, *p* < 0.0001), for cervicitis versus HSIL was 1.0000 (*p *< 0.0001) and for cervicitis versus CA was 1.0000 (*p* < 0.0001). AUC, Area Under Curve; ROC, Receiver Operating Characteristic.

**FIGURE 3:** The diagnostic ROC curve of the grayscale values of the small‐molecule probe for LISI versus HSIL and CA. The diagnostic AUC of the probe was 0.5484 (95% CI = 0.3826–0.7142, *p* = 0.5755) for LSIL versus HSIL and 0.7724 (95% CI = 0.6016–0.9432) for LSIL versus CA, *p* = 0.0138). AUC, Area Under Curve; ROC, Receiver Operating Characteristic.

**FIGURE 4:** The diagnostic ROC curve of the grayscale values of the small‐molecule probe for HSIL versus CA. The diagnostic AUC of the small‐molecule probe for HSIL versus CA was 0.7037 (95% CI = 0.4639–0.9435, *p* = 0.0896). AUC, Area Under Curve; ROC, Receiver Operating Characteristic.

### 3.3 Analysis of typical images

After comparing single probe images with merge images of different cervical lesion tissues, we found that the difference between groups was pronounced. Figure 5 shows a comparison of merge images of different cervical lesions. Figure 6 shows a comparison of Probe images of different cervical lesions.

**FIGURE 5:** Comparison of merge images of different cervical lesions. (A) The cervicitis group. (B) The LSIL group. (C) The HSIL group. (D) The CA group.

**FIGURE 6:** Comparison of Probe images of different cervical lesions. (A) The cervicitis group. (B) The LSIL group. (C) The HSIL group. (D) The CA group.

## 4 Discussion

In recent years, with the change in the lifestyle and dietary structure of residents, cervical cancer has shown a tendency toward rejuvenation, which brings a greater threat to women's physical and mental health [10]. Early accurate diagnosis is the premise of timely intervention and an important basis for improving the prognosis of patients with cervical cancer. At present, the methods for the diagnosis of cervical cancer include pathological detection, imaging examination, biochemical detection, biological genetic testing, and so forth, of which pathological detection and genetic testing have a long cycle, expensive cost, and are not suitable for clinical promotion. Biochemical detection is greatly affected by individual hormone levels and there may be remarkable variances before and after detection, imaging detection is easily affected by other organs of individuals, and biological genetic testing has the advantages of good reproducibility and high accuracy, so it has been popularized and applied in clinical practice [11, 12].

DNA methylation, specifically the methylation of 1 cytosine–phosphate–guanine dinucleotide, is an important epigenetic modification mechanism, and there is universal hypomethylation of the genome as well as hypermethylation of local regions in tumor tissues [13, 14]. Mutations and aberrant methylation of tumor suppressor genes may lead to uncontrolled cell proliferation and ultimately the formation of malignant tumors [15], the only mechanism in some cases. Hypermethylation may run through the occurrence and development of cervical cancer, and has its specific change pattern, so a molecular diagnosis of cervical precancerous lesions can be considered by DNA methylation detection, laying a good foundation for the screening of cervical cancer and early diagnosis and healing [16, 17].

The screening value of the small‐molecule probe in methylation markers of cervical cancer was analyzed by including 81 cases of different cervical lesions. The results showed that the grayscale values of cervical cancer tissues were remarkably higher than those of LSIL and cervicitis tissues, and the grayscale values of HSIL tissues were remarkably higher than those of LSIL and cervicitis tissues in quantitative comparison, which suggested that the grayscale values of different cervical lesions tissues were remarkably different. A study of 94 patients with high‐risk HPV infection showed that the detection rate of PAX1 gene methylation was 0.0% in normal cervical tissues, 13.0% in low‐grade lesions, 29.6% in high‐grade lesions, and 100.0% in cervical cancer tissues [18]. Moreover, the quantitative level of PAX1 gene methylation in 121 cervical tissues showed that the quantitative level of PAX1 gene methylation was (4.92 ± 4.45)% in normal cervical tissues, (5.55 ± 5.05)% in the low‐grade lesion group, (10.21 ± 14.39)% in the high‐grade lesion group, and (41.97 ± 23.02)% in the cervical squamous cell carcinoma group [19]. The authors analyzed that hypermethylation has a specific pattern of changes in each stage of the occurrence and development of cervical cancer, while the inactivation of different tumor suppressor genes caused by promoter hypermethylation occurs at different stages, and the additive effect of epigenetic alterations plays an important role in the carcinogenesis from normal cervical tissues to inflammatory tissues to precancerous lesions [20, 21].

The grayscale values in differentiating different cervical lesions were further analyzed by plotting the ROC curve. The results suggested that the grayscale values had good diagnostic efficacy in differentiating cervicitis tissues from the LSIL, HSIL, and CA, and also in differentiating LSIL from CA, but poor efficacy in differentiating LSIL from HSIL, and HSIL from CA. The authors analyzed that LSIL and HSIL belonged to precancerous lesions, even if it was difficult to differentiate in imaging and laboratory tests, while the process of HSIL and CA tissues was short, and the differentiation was easy to appear in confusion [22]. In addition, there may be some reasons that there are few cases included in the text, or general data have an impact on the results. If large sample and multi‐center data can be included, it will help to enhance the accuracy of the data.

## 5 Conclusion

In conclusion, the small‐molecule probe may help identify inflammatory lesions, precancerous lesions, and cancerous lesions in the cervix, but the efficacy in distinguishing precancerous lesions from cervical cancer still requires improvement.

## Conflicts of Interest

The authors declare no conflicts of interest.

## Data Availability

The data supporting the results of this study are available from the corresponding author.
